The article "Deconstruction of Knee Cartilage Injury in Athletes Using MR Images Based on Artificial Intelligence Segmentation Algorithm" was retracted in 2023. Reasons: signs of a paper mill; compromised peer review; unreliable results or conclusions.

# Deconstruction of Knee Cartilage Injury in Athletes Using MR Images Based on Artificial Intelligence Segmentation Algorithm

**DOI:** 10.1155/2022/4165232

**Published:** 2022-09-27

**Authors:** Yuze Zhang, Hao Lian, Yinghai Liu

**Affiliations:** Shanxi University Physical Culture Institute, Taiyuan 030006, Shanxi, China

## Abstract

The knee joint is the second largest joint in the human body, with a wide range of functional activities and strong support for the human body. Moreover, the cartilage of the knee joint is hyaline cartilage, which is relatively brittle, so it is most vulnerable to trauma. In clinical work, the damage of articular cartilage is a disease with a high rate of orthopedic visits. In this paper, all the experimental group cases included in the observation were patients with acute articular cartilage injury or OA diagnosed by knee arthroscopy. All experimental groups and control groups did not have any strenuous exercise one day before MRI (magnetic resonance imaging), and they sat for 30 minutes before the examination. Conventional scanning sagittal FSE-T1WI, FSE-T2WI, FS-FSE-T1WI, FS-FSE-T2WI, FS-PDWI, and coronal FS-PDWI sequence. In the normal control group, after the *T*2 color map was generated in the workstation, the articular cartilage was divided on the midsagittal plane, and the patellar cartilage and tibial plateau were roughly divided into upper, middle, lower and anterior, middle, and posterior thirds. In order to ensure the maximum comparability of the results, an artificial intelligence segmentation algorithm is used to divide the region of interest equally, and the central part of each partition is selected as much as possible for measurement. The *T*2 values of the three partitions of each cartilage were measured one by one and averaged. For the comparison results of *T*2 value of cartilage in the same part: according to patellar cartilage, femoral cartilage, and tibial cartilage, the *P* values are 0.973, 0.150, and 0.525, respectively. Therefore, early detection and early treatment of articular cartilage injury are of great significance to the performance of athletes' competition level and the extension of sports life.

## 1. Introduction

With the development of modern science, the research on articular cartilage surgical repair technology including cartilage autograft technology is changing with each passing day. The superiority of MR in accurately evaluating the repair effect is extremely important. However, there are various diseases that cause articular cartilage damage, often involving various joints of the whole body. Often the cartilage damage is not a single knee cartilage damage, which also puts forward higher requirements for the application space of MR imaging. Although there are various methods for examining the changes in knee articular cartilage, MR examination is currently widely used in clinical practice. MR not only overcomes the subjectivity of the images obtained by ultrasound but also shows the cartilage structure more clearly than X-ray and CT, and is considered as one of the best noninvasive methods for knee joint examination. Its advantages are that it can perform multidirectional, multiplane imaging, display complete joints, good tissue contrast, and observe different angles of tissue through three-dimensional images, which is very accurate for the evaluation of bone, articular cartilage, and soft tissue. The development and parameter optimization of MR hardware and software has greatly improved the resolution of knee cartilage images.

The article "Deconstruction of Knee Cartilage Injury in Athletes Using MR Images Based on Artificial Intelligence Segmentation Algorithm" was retracted in 2023. Reasons: signs of a paper mill; compromised peer review; unreliable results or conclusions.

The most direct sign of early knee cartilage damage is prolonged *T*2 relaxation time. Leichtenberg et al. believed that 60% to 80% of knee osteoarthritis (OA) patients have knee instability, which was associated with pain and limited mobility [1]. Zhou believed that the knee joint is one of the most important joints in the human body [2]. Li et al. believed that compared with walking and jogging, practicing TC may reduce the risk of knee injury [3]. Zhu et al. investigated 3D-DESS at different flip angles to evaluate 6 cartilage regions in each patient [4]. Nakamachi et al. believed that the articular cartilage of the knee has multiple functions, including dispersing stress in the tissue and absorbing shock [5]. However, the knee cartilage injury they proposed is only in research, and there is no good treatment plan. This paper will introduce an artificial intelligence segmentation algorithm to optimize it.

The artificial intelligence segmentation algorithm can ideally segment the femoral cartilage image. Rubini et al. proposed an unsupervised retinal vessel segmentation method based on contour detection [6]. Marczak et al. extended the practice of user-centric game testing to quantify user experience [7]. Wu et al. believed that Doppler optical coherence tomography (OCT) imaging of blood vessels after anastomosis can simultaneously provide high-resolution structure and blood flow imaging of blood vessels [8]. Padmavathi and Thangadurai used the color feature of the leaf image to segment the leaf image into multiple parts by color [9]. Kumar et al. proposed a new remote sensing hyperspectral scene segmentation technique [10]. But their proposed AI segmentation algorithm is not accurate enough.

In this paper, the clinical value of automatic cartilage segmentation software was evaluated by evaluating the contour of knee articular cartilage and calculating the error rate with the value obtained by radiologists segmenting articular cartilage as the gold standard. In this experiment, the sequence selection combined with the characteristics of the laboratory equipment, using the dominant sequence 3D-FS-FISP sequence showing cartilage morphology. At the same time, the double echo sequence was used to measure the *T*2 value of the cartilage signal, and the cartilage contour and signal abnormalities in patients with knee arthritis were evaluated by the combined application of the two sequences, and the data reflected the repair of cartilage damage after drug treatment. The differences in cartilage thickness and signal changes were evaluated by MR imaging, which fully affirmed the application value of the combined use of the two sequences in clinical research. The accurate segmentation of knee cartilage injury images based on MR can further assist doctors in evaluating the treatment response to related diseases, thereby providing a reliable basis for clinical diagnosis and treatment, formulation of rehabilitation strategies, and surgical planning. The purpose of image segmentation of knee cartilage injury is to divide the lesion area in the original 2D or 3D magnetic resonance image and use the mathematical algorithm of feature extraction, modeling, and measurement to extract and calculate accurate and repeatable pathological information, such as the maximum diameter, volume, and surface area of the lesions, so as to quantify the dynamic changes of the lesions in time and space before and after treatment. The study found that compared with arthroscopy and surgery, 23 patients (92%) had a positive rate and 3 patients had a negative arthroscopic examination (60%).

The article "Deconstruction of Knee Cartilage Injury in Athletes Using MR Images Based on Artificial Intelligence Segmentation Algorithm" was retracted in 2023. Reasons: signs of a paper mill; compromised peer review; unreliable results or conclusions.

## 2. Deconstruction Method of Knee Cartilage Injury in Athletes

### 2.1. Knee Cartilage Injury

Knee osteoarthritis is mainly manifested as a series of changes in articular cartilage and subchondral bone, and the early stage is mainly cartilage changes. Articular cartilage is a well-differentiated avascular tissue with an abundant extracellular matrix, and the repair ability of mature articular cartilage is extremely limited. Nowadays, there are many examination methods to visualize cartilage, of which arthroscopy is regarded as the gold standard for diagnosing cartilage damage, but it is invasive, expensive, and not suitable for surgical intervention before the disease is clearly defined and in the early stage of the disease. At present, the auxiliary examination methods for noninvasive examination of articular cartilage include ultrasound, X-ray (which is one of the most effective methods for early clinical detection, early diagnosis, and differential diagnosis of certain diseases), CT, and MR. Patients with obvious symptoms of knee pain cannot tolerate prolonged examinations. Compared with the FLASH imaging sequence, the DESS sequence is three-dimensional volume imaging with thin slices. Knee articular cartilage covers the surface of the knee joint in an irregular curved surface, with a large area but a thin thickness. It is curvilinear in sagittal and coronal views, and the surrounding anatomical structures are complex, requiring MR images to have high spatial resolution and signal-to-noise ratio [11].

The article "Deconstruction of Knee Cartilage Injury in Athletes Using MR Images Based on Artificial Intelligence Segmentation Algorithm" was retracted in 2023. Reasons: signs of a paper mill; compromised peer review; unreliable results or conclusions.

Injuries that penetrate the subchondral bone are repaired by fibrous tissue, fibrocartilagelike tissue, or hyaline cartilagelike tissue. After the subchondral bone is penetrated, the mesenchymal cells in the medullary cells in the medullary cavity and the cartilage damage area have multidifferentiation potential and can differentiate and grow into the cartilage in the specific environment of the joint cavity.

Trauma, inflammation, and other physical and chemical factors can all cause the loss of collagen fibers in articular cartilage, and the increase of water content in the cartilage. As the disease progresses, there will be local cartilage loss, and even the subchondral bone is exposed. Therefore, MR changes after knee cartilage injury include abnormal articular cartilage signal, loss of smooth surface contour, and changes in articular cartilage thickness and volume. The MRI features of articular cartilage injury are different for different reasons. The articular cartilage defect caused by acute cartilage trauma has a sharp edge and an acute angle with the subchondral bone, and cartilage fragments free in the joint can often be found. Osteoarthritis and other cartilage degenerative diseases are characterized by multiple articular cartilage defects with rounded edges and obtuse angles with subchondral bone. Indirect signs are subchondral bone sclerosis, subchondral cystic degeneration, osteophytes, intra-articular loose bodies, etc. When the disease in the knee joint weight-bearing area is more serious, it can cause uneven stenosis of the knee joint space. In inflammatory lesions, the thinning of articular cartilage due to the decomposition of enzymes is more extensive and uniform [12].

### 2.2. MR Images

Articular cartilage cannot be displayed in conventional X-ray and CT images, and can only be indirectly judged by the widening of the joint space and the changes in surrounding bone and soft tissue, so the false-positive rate of conventional X-ray and CT examinations is as high as 20%–40%. Ultrasound can observe the surface of bone dynamically from multisection, multiangle, and color. Doppler ultrasound can show pathological changes in articular cartilage and bone, but MRI is still the standard. The 3D-DESS (three-dimensional double-echo steady state) sequence is not only a three-dimensional gradient echo sequence that can perform thin-slice scanning but also can be used to assess the thickness changes in knee cartilage morphology. In this sequence, cartilage showed a moderate signal, while joint fluid showed a high signal [13].

The article "Deconstruction of Knee Cartilage Injury in Athletes Using MR Images Based on Artificial Intelligence Segmentation Algorithm" was retracted in 2023. Reasons: signs of a paper mill; compromised peer review; unreliable results or conclusions.

The cases of knee cartilage injury treated in our hospital were collected, and preoperative MR imaging was performed on the patients, who planned to undergo knee arthroscopy, and there was no history of knee joint surgery. A total of 34 patients underwent knee arthroscopy within 2 weeks after MR examination. For the measurement of the specimens, the maximum diameter of the articular cartilage injury area was measured as the long diameter using a submeter, and the maximum diameter was measured in the vertical direction as the transverse diameter. Then use a vernier caliper to measure the distance between the feet of the subruler, the unit of measurement is mm, and the accuracy is 0.05 mm. In order to reduce the measurement error, each part was measured three times, and the average value was taken at last. The three-dimensional reconstruction of articular cartilage was carried out in two steps on the Advantage Workstation3.1 image workstation (its advanced visualization and diagnostic capabilities allow clinicians to share images quickly and easily). First, on the FS-3D-FISP sagittal image, the contour of the femoral condyle and articular cartilage on the surface of the trochlear surface was obtained by cutting layer by layer. It includes the adjacent tissues of part of the articular cartilage to avoid the influence of subjective factors on the morphology of the articular cartilage. Secondly, the appropriate threshold selection is performed on the reconstructed image of the articular cartilage surface including some adjacent tissues to remove the surrounding tissue images and reveal the surface morphology of the articular cartilage. Finally, the 3D reconstructed images of the articular cartilage were displayed in MIP (maximum density projection) mode. The 3D measurement was performed directly on the surface and MIP 3D reconstruction images of the articular cartilage. The maximum diameter of the articular cartilage damage area was measured as the long diameter, and then the maximum diameter was measured in the vertical direction as the transverse diameter. Each site was measured three times, and the average was taken at the end. The MRI examination is shown in Figure 1.

The article "Deconstruction of Knee Cartilage Injury in Athletes Using MR Images Based on Artificial Intelligence Segmentation Algorithm" was retracted in 2023. Reasons: signs of a paper mill; compromised peer review; unreliable results or conclusions.

Groups of healthy volunteers were used primarily for technical assessments. To exclude the influence of operators with different experiences and skills on the experiment, all volunteer MR examinations were scanned by the same person. During the examination, the volunteers were in the supine position with both feet in the advanced position. All examinations were performed on a clinical large-bore (70 cm diameter) whole-body 3T MRI scanner equipped with a dedicated eight-channel knee coil with a maximum gradient field strength of 45 mT/m and a maximum conversion rate of 200 mT/m. In addition to routine clinical scans, 3T MRI is also responsible for many advanced clinical examinations and scientific research work in hospitals. All subjects' knees were in the middle of the coil and used consistent spatial positioning. Several small pillows were placed around the knee joint to reduce coil motion artifacts [14].

The 3D source image can be reconstructed in coronal, sagittal, and axial directions (coronal view: parallel to the femoral condyle; sagittal view: along the anterior cruciate ligament (ACL); axial view: perpendicular to the posterior cartilage of the patella), and the reconstruction is performed using 3D software on the siemens VERIO-WMMMP console, and the image reconstruction thickness is 0.6 mm. The signal-to-noise ratio (SNR) is the ratio of the signal intensities of the image and background random noise, the signal-to-noise ratios of six different cartilages of the medial and lateral femoral cartilage, medial and lateral tibial cartilage, trochlear cartilage and patellar cartilage were calculated, respectively. The formula for calculating the signal-to-noise ratio is [15]as follows:

(1) $$\begin{array}{c} \text{SNR}=\frac{\text{SI}}{\text{SD}}\times 100\text{\%}, \end{array}$$

(2) $$\begin{array}{c} \text{CNR}=\left|{\text{SNR}}_{\text{Structure}1}-{\text{SNR}}_{\text{Structure}2}\right|\times 100\text{\%}. \end{array}$$

Before arthroscopic exploration (through the incision of the skin hole, the camera and surgical instruments are extended into the joint, and under the monitoring of the monitor, the doctor operates to diagnose and treat various joint diseases), two physicians jointly read the films and made a diagnosis of the cartilage in each sequence of images and a diagnosis of the lesion grade. The grade is based on the most obvious articular cartilage damage. The cartilage was divided into 5 grades according to Recht classification and Outerbridge classification by arthroscopy. Microsoft Office Excel 2007 office software and SPSS V18.0 were used for data entry and analysis of cartilage, joint fluid, background SNR, and CNR of cartilage and joint fluid scanned under different FAs by 3D-DESS sequence. The Bonferroni method (it is the method used to control the overall confidence level of a whole set of confidence intervals) was used to correct the data of multiple repeated measures, and the general standard linear mixed model statistical analysis, *p* < 0.05 was statistically significant. The FA corresponding to the highest CNR of cartilage and joint fluid is a set of sequences optimized for 3D-DESS [16].

The article "Deconstruction of Knee Cartilage Injury in Athletes Using MR Images Based on Artificial Intelligence Segmentation Algorithm" was retracted in 2023. Reasons: signs of a paper mill; compromised peer review; unreliable results or conclusions.

During the imaging process of MRI images, due to the influence of other factors, noise is inevitably generated, which also affects the accuracy of segmentation to a certain extent. Let the observed image be *Y*, the real image be *X*, and the offset field is *B*. Then for each pixel *i* there is [17]as follows:

(3) $$\begin{array}{c} Y=X_{i}B. \end{array}$$

Perform ln conversion to get [18]:

(4) $$\begin{array}{c} y=x_{i+}\theta \beta_{i}. \end{array}$$

For a given *Y* or *y*, how to get *X* accurately is the focus of current research [19].

Since the BP algorithm only uses the grayscale information (the thumbnails of the red, green, and blue channels are all displayed in grayscale) of the image pixels without considering the spatial information, the offset field and noise will change the value of the membership matrix, which will cause the wrong classification of some pixels during image segmentation, which will ultimately affect the segmentation results. For such a situation, this paper proposes an improved artificial intelligence segmentation algorithm for image segmentation. This method incorporates the neighborhood information of pixels into the solution of the clustering criterion function value, and the improvement is as follows [20]:

(5) $$\begin{array}{c} J\left(A,V\right)=\sum^{}\sum^{}a\left|x-v\right|+\frac{a}{n}\sum^{}\sum^{}\left(x-v\right). \end{array}$$

Among them, *a* is the influence factor of the neighborhood on the clustering criterion function, which is affected by the signal-to-noise ratio (SNR) of the image, and a lower SNR value determines a higher a, and vice versa. To achieve the minimum value, the Lagrangian multiplication factor is introduced, let [21]:

(6) $$\begin{array}{c} Fm=\sum^{}\sum^{}\left(aD+\frac{\sigma }{n}\right)+\gamma \sum^{}\sum^{}\left(y-\beta -v\right). \end{array}$$

Among them:

(7) $$\begin{array}{c} D=y-\beta -v, \end{array}$$

(8) $$\begin{array}{c} \gamma =\sum^{}y-\beta -v^{2}. \end{array}$$

Derivation in the direction, while making its value 0, get [22]:

(9) $$\begin{array}{c} \frac{\partial Fm}{\partial aij}=maD+\frac{\alpha m}{N}a=0. \end{array}$$

### 2.3. Artificial Intelligence Segmentation Algorithm

The spatial structure of knee cartilage injury images is highly complex, and the artifacts in the MRI imaging process lead to the internal variability of the pixel gray levels of each tissue. After preprocessing, a single Gaussian model can well model the grayscale changes with obvious differences, so as to realize the segmentation of relatively fixed tissues or organs. However, since GMM (adaptive background mixture models for real-time tracking) does not consider any spatial factors in modeling, it is difficult to directly model the complex damage area with variable size and location. Therefore, GMM is often used for presegmentation of surrounding tissue or lesion area in damaged images, and its segmentation results can be used as prior knowledge, combined with other features such as the shape and appearance of the lesion, to continue training the model to optimize the segmentation.

The article "Deconstruction of Knee Cartilage Injury in Athletes Using MR Images Based on Artificial Intelligence Segmentation Algorithm" was retracted in 2023. Reasons: signs of a paper mill; compromised peer review; unreliable results or conclusions.

Early detection and diagnosis of articular cartilage damage are of great significance for timely clinical intervention and treatment. With the help of artificial intelligence-assisted software, three-dimensional parameters such as cartilage *T*2, *T*2^*∗*^, and other biochemical indicators and volume can be directly obtained, which greatly improves the accuracy and utilization of data. The development of MRI, such as three-dimensional quantitative magnetic resonance imaging, allows for a more sensitive analysis of cartilage morphology. Using high-resolution 3D MRI sequences and automated cartilage segmentation software, cartilage quantitative parameters such as cartilage volume and thickness can be obtained noninvasively. In the evaluation of articular cartilage and cartilage repair tissue, *T*2^*∗*^ relaxation (magnetization in the transverse direction) parameters showed a certain change law. These morphological and biochemical imaging indicators can be obtained through the software, which can quantitatively evaluate cartilage and greatly save postprocessing time. Therefore, these tools have certain application value in clinical practice. However, the automatic segmentation software has certain errors in the segmentation of cartilage subregions. The image segmentation process is shown in Figure 2. Preprocessing can reduce the artifacts in the image to enhance the image quality; segmentation is to divide the pixels into different regions, and defines the boundaries of different tissues.

In image segmentation, GMM can be used to cluster pixels into multiclass labels. For a given image *X*, GMM calculates the probability distribution at each pixel *x*, as *M* Gaussian components, as follows [23]:

(10) $$\begin{array}{c} f\left(x\right)=\sum^{}wn\left({\text{sin}}^{-1}x,\sigma_{i}^{2}\right). \end{array}$$

The CRF model (the two adjacent hidden states are related, but not who depends on whom) has been widely used in the regularization of medical image segmentation results. Because the size, shape, and position of the lesion area in medical images are usually unpredictable, it is difficult to model it directly, and CRF can directly constrain the segmentation results based on the neighborhood information. However, because the traditional CRF often only considers the constraints between adjacent pixels, the modeling of global information is not sufficient, and it is easy to converge to a local minimum in the optimization process of the energy potential function. Therefore, the segmentation results for regions with relatively blurred boundaries are not satisfactory.

The article "Deconstruction of Knee Cartilage Injury in Athletes Using MR Images Based on Artificial Intelligence Segmentation Algorithm" was retracted in 2023. Reasons: signs of a paper mill; compromised peer review; unreliable results or conclusions.

Similar to CRF, automatic context also needs to solve the maximum posterior probability, which mainly focuses on the marginal distribution:

(11) $$\begin{array}{c} f\left(x\right)=\sum^{}wn\left({\text{sin}}^{-1}x,\sigma_{i}^{2}\right). \end{array}$$

In order to make full use of more context information to better approximate the posterior distribution of the objective function, the automatic context model uses the segmentation probability map obtained by the traditional classifier to construct a new training set. Specifically, by feeding the training set into the trained classifier, a segmentation probability map can be obtained, which is added as one of the features of the new training set:

(12) $$\begin{array}{c} \varphi =\left\{\text{y},f\left(x\right),p^{0}\left(i\right)\right\},i=1,2,\cdots ,n. \end{array}$$

Among them, *p*^0^ represents the initial probability map corresponding to the training image, and *p*^0(*i*)^ represents the probability value centered on the *i*th pixel obtained from the training data.

This paper mainly selects several evaluation indicators:

(1) The Dice coefficient is used to describe the volume overlap between the segmentation result and the gold standard. The larger the Dice, the more similar the segmentation result is to the gold standard.
  (13) $$\begin{array}{c} D\left(Y,\hat{Y}\right)=\frac{2\left|Y\cap^{}\hat{Y}\right|}{\theta \left|Y\cap^{}\hat{X}\right|}. \end{array}$$
(2) Precision, which means that among the voxels classified as target lesions in the segmentation results, the proportion of voxels that actually target lesions; the higher the precision, the more accurate the segmentation.
  (14) $$\begin{array}{c} P\left(Y,\hat{Y}\right)=\frac{\text{N}\left|Y\cap^{}\hat{Y}\right|}{\left|Y_{1}\cap^{}\hat{Y}\right|}. \end{array}$$
(3) Specificity, which indicates the proportion of voxels classified as nontarget lesions in the segmentation results among all the voxels that are actually nontarget lesions.
  (15) $$\begin{array}{c} \text{Specificity}\left(Y,\hat{Y}\right)=\frac{N\left|Y_{0}\cap^{}\bar{Y_{0}}\right|}{\left|Y_{0}\right|}. \end{array}$$
(4) Sensitivity, which indicates the proportion of voxels classified as target lesions in the segmentation results among all the voxels that actually target lesions; the higher the sensitivity, the more comprehensive the segmentation.
  (16) $$\begin{array}{c} \text{Sensitivity}\left(Y,\hat{Y}\right)=\frac{\left|Y_{1}\cap^{}\bar{Y_{1}}\right|}{\left|Y_{1}\right|}. \end{array}$$

The high-dimensional feature set corresponding to the training image is denoted as *f*(*X*, *A*), where *A* represents the image set from different modalities and *f* represents the feature set. After inputting the image into the traditional random forest model, the final segmentation result can be expressed as:

(17) $$\begin{array}{c} P\left(Y|X\right)=\frac{1}{T}\sum^{}\left(\sigma +f\left(X,A\right)\right). \end{array}$$

Assuming that the voxel gray distribution of the input image is a fixed condition, the total energy function is as follows:

(18) $$\begin{array}{c} E\left(Y\right)=\epsilon \sum^{}\rho \left(y\right)+\sum^{}\varphi \left(y\right). \end{array}$$

The article "Deconstruction of Knee Cartilage Injury in Athletes Using MR Images Based on Artificial Intelligence Segmentation Algorithm" was retracted in 2023. Reasons: signs of a paper mill; compromised peer review; unreliable results or conclusions.

### 2.4. Statistical Processing

*T* values for 15 regions of interest were obtained for each patellar cartilage measurement, and the average patellar cartilage *T*2 values were obtained by averaging these 15 *T*2 values as:

(19) $$\begin{array}{c} T2\text{av}=\frac{\left(T_{2}1+T_{2}2+T_{2}3+\cdots +T_{2}15\right)}{15}. \end{array}$$

Similarly, each patellar cartilage is divided into 5 regions, and the average *T*2 value for the lateral region is obtained by averaging the three levels:

(20) $$\begin{array}{c} \text{outerzone}T2\text{av}=\frac{\left(T_{2}1\text{outerzone}+T_{2}2\text{outerzone}+T_{2}3\text{outerzone}\right)}{3}. \end{array}$$

The average *T*2 values of the other 4 regions of the patellar cartilage (*T*2av lateral, *T*2av central, *T*2av medial, and *T*2av medial) were calculated in a similar way to the lateral region.

SPSS16.0 software package was used for the following statistical processing, and *P* < 0.05 was considered to be statistically significant.

1. The paired samples *t* test was used to analyze the difference between the average *T*2 value (*T*2av) of the bilateral patellar cartilage in hockey players and the difference in the average *T*2 value of the bilateral patellar cartilage (*T*2av) in healthy volunteers.
2. Two-sample *t* test was used to analyze the *T*2 value of the right knee cartilage in the two groups (athletes and healthy volunteers), and the difference in the *T*2 value of the left knee patellar cartilage between the two groups (hockey players and healthy volunteers).

The article "Deconstruction of Knee Cartilage Injury in Athletes Using MR Images Based on Artificial Intelligence Segmentation Algorithm" was retracted in 2023. Reasons: signs of a paper mill; compromised peer review; unreliable results or conclusions.

## 3. Evaluation Results of Knee Cartilage Injury in Athletes

Among the 30 patients, there were 60 cartilage injuries, of which the cartilage surface was smooth, and 8 spots or small pieces of abnormal signals were seen inside. The remaining 52 places showed changes in the shape of cartilage, including 17 cartilage surface imperfections, depressions, and partial cartilage defects but less than 1/2 of the full thickness. The cartilage defect reached more than 1/2 of the full thickness, but the bone was not exposed, and the surface was rough and not smooth in 16 places. The differences in BIM (body mass index) are shown in Table 1.

A total of 38 cartilage injuries in 20 patients were selected. The surface of cartilage was smooth, the three-layer structure of cartilage was not clear, and there were 7 spots or small pieces of abnormal signal, which were low signal in 3D-FS-SPGR sequence, and unclear in 3D-FIESTA sequence. The remaining 31 places were all manifested as cartilage morphological changes. Among them, the contour of cartilage was irregular, localized thinning, partial or most defects of cartilage, rough surface, and 26 spots; 5 spots of full-thickness cartilage exfoliation. The ICC test results are shown in Table 2.

Of the thirty patients: 5 patients (16.6%) had normal MRI appearance. MRI found 25 patients (83.4%) with knee injury, 15 of the 25 patients had knee injury, (60%) had ACL injury, 2 patients (8%) had PCL injury, 10 cases (40%) had meniscus injury, 8 cases (32%) had collateral ligament injury in 5 cases (20%), and bone injury in 2 cases (8%). Only 7 (28%) were isolated injuries, while 18 (72%) were complex injuries. Compared with arthroscopy and surgery, the positive rate was positive in 23 of 25 patients (92%), and 3 out of 5 patients with negative MRI findings were negative by arthroscopy (60%). Morphological analysis showed an overall sensitivity of 92% and specificity of 60%. For 15 cases of ACL injury, 13 cases (88.4%) were true positive in 8 cases (82%), and 10 cases with meniscus injury were truly positive. The advantage of MRI in knee injury is that MRI can be used for knee joint examination in the early stage of injury or after trauma, MRI can detect a variety of problems such as: meniscus tears, ligament tears, bone contusions, osteochondral defects, and can also detect less common conditions. The characteristics of magnetic resonance imaging in different injured parts of the knee joint are shown in Table 3.

The *T*2 values of the lateral and lateral areas of the right patellar cartilage (*T*2av lateral area, *T*2av lateral area) were higher than those of the left patellar cartilage. The range of the right patellar cartilage *T*2av lateral area is 39.25–55.01 (ms) and the average is 43.55 ± 5.38 (ms). The range of the right patellar cartilage *T*2av lateral area was 36.87–47.28 (ms), and the mean value was 42.66 ± 5.09 (ms). The range of the left patellar cartilage *T*2av lateral area was 35.26–43.67 (ms), the mean value was 41.33 ± 4.39 (ms), and the left patellar cartilage *T*2av lateral area range was 35.75–44.54 (ms), the mean value was 41.22 ± 4.11 (ms). The *T*2 value in the lateral area of *T*2av is 2.41 (ms) higher on the right side than the left side on average, and the *T*2 value on the right side is 1.82 (ms) higher than the left side on the lateral area of *T*2av. The paired sample *t* test showed that there were significant differences between the groups in the lateral region of *T*2av (*t* = 2.51, *P* = 0.02) and the lateral region of *T*2av (*t* = 2.29, *P* = 0.04). Although the *T*2 values of the medial, medial, and central areas of the left patellar cartilage (*T*2av medial, *T*2av medial, and *T*2av central) were slightly higher than those of the left patellar cartilage, by paired sample *t* test, the difference was not statistically significant (*P* > 0.05).  Table 4 shows the different degrees of injury in the left and right patellar cartilage regions of athletes.

The article "Deconstruction of Knee Cartilage Injury in Athletes Using MR Images Based on Artificial Intelligence Segmentation Algorithm" was retracted in 2023. Reasons: signs of a paper mill; compromised peer review; unreliable results or conclusions.

When the cartilage is severely damaged, it is not difficult to identify the cause of the damage according to the morphological changes of the cartilage. However, when the cartilage is mildly damaged, it is difficult to identify acute and chronic cartilage damage based solely on changes in cartilage signals, and it is often necessary to combine other changes in the joint. For example, bone contusion and fracture are common symptoms of acute injury. However, when the cartilage is mildly damaged, it is difficult to identify acute and chronic cartilage damage based solely on changes in cartilage signals, and it is often necessary to combine other changes in the joint. For example, bone contusion and fracture are common symptoms of acute injury. Moreover, the lesions of cartilage damage often correspond to the sclerotic lesions of the subchondral bone, multiple lesions are common, and there are generally no signs of cartilage and bone fractures. MRI is far less accurate than arthroscopy in showing cartilage contour damage and is also affected by many external conditions such as patient age, body position, volume effect, magic angle effect, examination sequence, and imaging orientation.

In order to verify the effectiveness of artificial intelligence segmentation algorithm for MR knee femoral cartilage segmentation, we will use the classical figure cut algorithm as a control. Ten MR knee images with different image sequences and different slice positions were selected as experimental materials. Eight independent femoral cartilage segmentation operations were performed on each image by applying the algorithm in this paper and the classical figure cut algorithm. And in each segmentation, the manual interaction of these two algorithms is the same, that is, the selected seed pixels are the same. The parameters of the algorithm in this paper are set to 5. For the parameters of the classical figure cut algorithm, after many experiments, a set of configurations with the best comprehensive effect is selected: the potential energy coefficient is 0.5, and the variance parameter is 14. The segmentation effect of the algorithm in this paper is indeed better than that of the classical figure cut algorithm. The segmentation results of the latter often show some discrete incorrect blocks in the background area. The algorithm in this paper almost never happens. Moreover, the classical figure-cut algorithm often cannot segment the target image as a whole, but the algorithm in this paper is more ideal in this respect. Since the image of femoral cartilage is narrow in shape and very similar to the image of some surrounding tissues, this is a major problem in femoral cartilage segmentation. The effectiveness of artificial intelligence segmentation algorithm for MR knee femoral cartilage segmentation is shown in Figure 3. For some femoral cartilage section images with narrow shapes, the segmentation error of the classical figure cut algorithm is relatively large. Only for some relatively thick parts, the segmentation task can be barely completed. The algorithm in this paper can achieve the basic segmentation requirements for the segmentation of femoral cartilage images in all parts. Although the DSC value of the segmentation results is low for some cartilage images in some sections, the basic contour of the target cartilage can still be segmented. Compared with the classical figure cut algorithm, the DSC value of the segmentation results obtained by the artificial intelligence segmentation algorithm is increased by 70% on average. The experimental results show that the proposed algorithm is effective for the segmentation of MR knee femoral cartilage images.

The article "Deconstruction of Knee Cartilage Injury in Athletes Using MR Images Based on Artificial Intelligence Segmentation Algorithm" was retracted in 2023. Reasons: signs of a paper mill; compromised peer review; unreliable results or conclusions.

There were 30 left patellar cartilages (26 in the sports trauma group and 24 in the control group). The average *T*2 value (*T*2av) of the left patellar cartilage in the sports trauma group was also higher than that in the control group. The average *T*2 value (*T*2av) of the left patellar cartilage in the sports trauma group ranged from 35.38 to 42.38 (ms), with an average value of 38.82 ± 4.68 (ms). The average *T*2 value (*T*2av) of the left patellar cartilage in the control group ranged from 32.62 to 36.52 (ms), with an average value of 35.32 ± 3.86 (ms). After the two-sample *t*-test, it cannot be considered that the variance between the two groups is not equal (*F* = 2.58, *P* = 0.22), and there is a significant difference between the groups (*t* = 6.82, *P* = 0.0005). The comparison of the average *T*2 value (*T*2av) of the left and right patellar cartilage in the sports trauma group and the control group is shown in Table 5.

Whether it is acute trauma or articular cartilage damage caused by OA, changes in cartilage appearance will occur. The control group included 14 cases with 28 patellar cartilages. Its *T*2 value is also detailed in Tables 2 and 3. The average *T*2 value (*T*2av) of the right patellar cartilage ranged from 32.79 to 37.76 (ms), and the mean value was 35.60 ± 4.26 (ms). The average *T*2 value (*T*2av) of the left patellar cartilage ranged from 32.71 to 37.52 (ms), and the mean value was 35.01 ± 3.87 (ms). The average *T*2 value (*T*2av) of the right patellar cartilage was slightly higher than that of the left patellar cartilage. The paired sample's *t* test showed *t* = 1.47, *P* = 0.16 (*P* > 0.05), and there was no significant difference. The average *T*2 value of 28 patellar cartilages (420 small ROIs in total) in healthy volunteers was 35.31 (ms). Considering the low average value, this paper takes 110% of the average *T*2 value of the left and right knee cartilage of all healthy volunteers as the reference threshold for judging whether the cartilage is damaged. That is, 38.84 (ms), which is close to the upper limit of the average *T*2 value of the patellar cartilage in healthy volunteers, that is, if it is higher than this value, it is judged as injury, which can be used as a reference for estimating the degree of patellar cartilage injury in athletes below. The mean *T*2 values of the subjects' bilateral patellar cartilages are shown in Figure 4.

The *T*2-map in the mild cartilage injury group showed that the articular cartilage was continuous, but the joint space was not narrow. The *T*2 value of mildly injured articular cartilage in the acute trauma group ranged from 40.62 to 58.32 ms, with an average of (50.85 ± 4.70) ms. In the severe cartilage injury group, the *T*2-mapping color map was interrupted or incomplete. In the OA group, the *T*2 value of the severely injured articular cartilage ranged from 41.89 to 59.76 ms, with an average of (51.22 ± 4.66) ms. According to the comparison of mild injury, severe injury, the severity of OA (osteoarthritis), and the severity of acute trauma, the *P* values were 0.788, 0.404, 0.507, and 0.352. The comparison of percent error of surface 3D measurement of lesions with different damage degrees is shown in Figure 5.

The article "Deconstruction of Knee Cartilage Injury in Athletes Using MR Images Based on Artificial Intelligence Segmentation Algorithm" was retracted in 2023. Reasons: signs of a paper mill; compromised peer review; unreliable results or conclusions.

There were statistically significant differences in the injury time (*P* = 0.002 < 0.05), the number of repeated sprains of the knee joint (*P* = 0.000 < 0.05), and the preoperative Lysholm score (*P* = 0.005 < 0.05) between the two groups. The injury time of group *B* (with cartilage damage) was significantly longer than that of group *A* (without cartilage damage), and the number of repeated knee sprains in group *B* was significantly more than that in group *A*. It shows that the longer the course of the disease, the higher the proportion of patients with unstable reinjury history. The preoperative Lysholm score of group *B* patients was significantly higher than that of group *A* patients, considering that most patients in group *A* had a shorter course of the disease, and suffered from obvious symptoms such as knee joint swelling, limited activity, and low activity. The preoperative Lysholm score is shown in Table 6.

Cartilage surface is smooth, swollen, abnormal color, or soft to the touch in 14 places. Irregular bone surface, surface linelike fissures, or craterlike defects, and the thickness of the defect is less than 1/2 of the full thickness of cartilage in 28 places. The surface of the cartilage is uneven or has crablike changes and the thickness of the defect is greater than 1/2 of the full thickness, but the subchondral bone has not been exposed in 32 places. Full-thickness cartilage defect and 26 exposed subchondral bone. The severity of lesions on MRI examinations is shown in Figure 6. I–IV are arthroscopic diagnostic grades.

The total number of lesions for each grade assessed by MRI was arthroscopically assessed as a percentage of that grade. And drawn into a figure, the *x*-axis represents the coincidence rate of each grade of MRI, the *y*-axis represents the grade of cartilage damage assessed by MRI, and the top straight line represents the 100% coincidence rate. The higher the curve is, the closer it is to the preset line, indicating that the sequence has a higher coincidence rate for the classification of chronic knee joint injury, and the evaluation results are more credible. The average coincidence rate of FS-3D-SPGR was the highest, and the coincidence rates among the grades were similar. The average coincidence rate of SE-T1WI was the smallest and the coincidence rate between grades varied greatly. The grading coincidence rate of MRI for cartilage damage is shown in Figure 7.

The article "Deconstruction of Knee Cartilage Injury in Athletes Using MR Images Based on Artificial Intelligence Segmentation Algorithm" was retracted in 2023. Reasons: signs of a paper mill; compromised peer review; unreliable results or conclusions.

The contrast-to-noise ratio (CNR) of cartilage to surrounding tissue in different sequences is shown in Figure 8. The 3D-FIESTA sequence belongs to the gradient echo sequence, and its main feature is that its repetition time (time of repetition, TR) is extremely short, so the imaging speed is very fast, and it can provide a high signal-to-noise ratio. When this sequence is used for knee joint examination, the signal of cartilage is low, and the signal of surrounding bone is slightly high, which improves the contrast between the two. Secondly, the three-dimensional Fourier transform recombination acquisition method applied in this sequence can obtain images with thin layers, high signal-to-noise ratio, and high resolution. The 3D-FIESTA image can also create a better contrast between the synovial fluid and cartilage signals and is more sensitive to the display of bone marrow edema or bone contusion, which is more conducive to the detection of cartilage damage. The signal of the fluid and fat-rich bone marrow in the knee joint decreased significantly, so in the knee joint imaging, the articular cartilage became the only high signal structure, and the contrast between the articular cartilage and the adjacent tissues was significantly improved. In the past, some scholars suggested that the long scanning time was the disadvantage of this sequence. In this paper, the number of excitations (NEX) was changed to 1, which significantly shortened the scanning time. Comparing the application of the two in knee cartilage lesions, both can better show the damage to articular cartilage. In the 3D-FIESTA sequence, the subchondral bone lesions are mostly low signal, while the bone itself is a slightly high signal, while in 3D-FS-SPGR, the low signal of the bone itself conceals part of the intraosseous lesions, the lesion range is smaller than that of the 3D-FIESTA sequence. Therefore, the sensitivity of 3D-FIESTA sequence in showing bone lesions is higher than that of 3D-FS-SPGR sequence. The damage to cartilage is often accompanied by abnormal subchondral bone signals. Therefore, in the display of articular cartilage lesions, the combined observation of the two sequences is more conducive to the detection of lesions.

The subchondral bone and the fluid in the joint cavity showed low signal, while the cartilage showed high signal, which constituted an obvious signal gradient, and the intrachondral lesions were clearly displayed. On the 3D-FIESTA sequence, the articular cartilage showed a less clear layered structure and an obvious band-like low signal. The subchondral bone lesions are more clearly displayed in this sequence, and the range is more comprehensive than that displayed by 3D-FS-SPGR sequence, which is manifested as a low signal with unclear boundary. The Kappa value of 3D-FS-SPGR sequence was 0.732 (>0.60), which was 78.4% completely consistent with the results of arthroscopy. The sensitivity and specificity of the 3D-FIESTA sequence were 82% and 88.7%, respectively, and the Kappa value was 0.708 (>0.60). The complete agreement with the results of arthroscopy was 76.4%, and there was no significant difference in the agreement between the two sequences (*χ*^2^ = 0.286, *P* = 0.593). The comparison of sensitivity and specificity is shown in Figure 9.

The article "Deconstruction of Knee Cartilage Injury in Athletes Using MR Images Based on Artificial Intelligence Segmentation Algorithm" was retracted in 2023. Reasons: signs of a paper mill; compromised peer review; unreliable results or conclusions.

In the early stage of OA, the synthesis and decomposition of cartilage ECM are unbalanced, the collagen on the cartilage surface is degenerated, degenerated, destroyed, and the morphology and arrangement of collagen fibers are abnormal. These biochemical changes cause cartilage damage. At the same time, the synthesis of PGs is inhibited and lost, and the expansion and contraction space of the remaining PGs will be significantly increased. At the same time, the frictional resistance of water decreases, and the final result of the dual action is the increase of water content in the cartilage. The most direct imaging manifestation is the prolongation of *T*2 relaxation time. The increase of water content in cartilage, the destruction of the collagen network, and the reduction of PGs all significantly reduced the liquid pressure of cartilage, weakened the cartilage's carrying capacity, and eventually led to cartilage exfoliation and loss of its proper function. That is to say, the *T*2 value of articular cartilage can be measured to evaluate whether it is damaged or not. Based on this, the *T*2-mapping sequence came into being.

Taking the results of arthroscopic grading diagnosis as the standard, the normal control group and acute trauma group were measured in ADW4.4 workstation of MRI, respectively. The three-layer structure of cartilage can be seen in the Tz-map color map of a normal knee joint, the surface layer is green, the middle layer is yellow, and the inner layer is green. The average *T*2 value of patellar cartilage was (36.94 ± 3.10) ms, the *T*2 value of femoral cartilage was 35.18–47.74 ms, the average was (41.83 ± 3.22) ms, and the *T*2 value of tibial cartilage was 34.21–50.76 ms, the average was (42.61 ± 4.85) ms. In the acute trauma group, the range of *T*2 value of patellar cartilage was 40.62–50.76 ms, the average was (45.95 ± 3.72) ms, the range of *T*2 value of femoral cartilage was 46.90–58.32 ms, the average of (52.18 ± 3,73) ms, the range of *T*2 value of tibial cartilage was 46.66–58.67 ms, the average was (53.57 ± 3.34) ms. In group 0A, the *T*2 value of the patellar cartilage ranged from 41.38 to 51.20 ms, with an average of (46.01 ± 3.88) ms, and the *T*2 value of the femoral cartilage ranged from 40.75 to 56.85 ms, with an average of (50.43 ± 3.94) ms. The *T*2 value of tibial cartilage ranged from 46.83 to 59.76 ms, with an average of (52.75 ± 4.13) ms. The average *T*2 value of articular cartilage in the same part of the acute trauma group and OA group was higher than the average *T*2 value of normal articular cartilage in the corresponding part, and the *T*2 value of cartilage in the same part was compared. Arranged by patellar cartilage, femoral cartilage, and tibial cartilage, the *P* values were 0.973, 0.150, and 0.525. A comparison of cartilage *T*2 values is shown in Figure 10.

The article "Deconstruction of Knee Cartilage Injury in Athletes Using MR Images Based on Artificial Intelligence Segmentation Algorithm" was retracted in 2023. Reasons: signs of a paper mill; compromised peer review; unreliable results or conclusions.

## 4. Conclusions

With the application and development of MRI technology in clinical work, the conventional sequences also have certain limitations in the display of cartilage lesions. Therefore, this paper retrospectively analyzed the imaging manifestations of cartilage injury caused by pure acute trauma and pure chronic cartilage injury, in order to find out whether there is any difference in the imaging manifestations of the two. At the same time, the three unconventional sequences were compared, and the artificial intelligence segmentation algorithm was used to find the most valuable image sequence showing articular cartilage lesions. In this paper, the results of arthroscopy were taken as the basic criteria, and the chi-square test was used to compare the diagnostic results of 3D-FIESTA and 3D-FS-SPGR MRI sequences and the comparison of their consistency in the detection of lesions. Using the measurement result of *T*2 value as the original data, the difference of each observation value among the acute trauma group, OA group, and control group and the difference in the observation value of patellar cartilage, femoral cartilage, and tibial cartilage in each group were analyzed. Combined with the grading standard of articular cartilage injury, the injury was defined as a mild injury and severe injury, and the grading results of arthroscopy were used as the standard to analyze the difference in *T*2 value between mild injury, severe injury, and normal control group. In future work, MRI and arthroscopy can be performed at the same time to more accurately estimate cartilage damage, including damage level grading, damaged area, etc. [24, 25].

## Figures and Tables

**Figure 1:** MRI examination.

**Figure 2:** Image segmentation process.

**Figure 3:** Effectiveness of artificial intelligence segmentation algorithm for MR knee femoral cartilage segmentation.

**Figure 4:** The mean *T*2 value of the subject's bilateral patellar cartilage.

The article "Deconstruction of Knee Cartilage Injury in Athletes Using MR Images Based on Artificial Intelligence Segmentation Algorithm" was retracted in 2023. Reasons: signs of a paper mill; compromised peer review; unreliable results or conclusions.

**Figure 5:** Comparison of percent error of surface 3D measurement for lesions with the same degree of damage.

**Figure 6:** Severity of lesions on MRI.

**Figure 7:** The grading coincidence rate of MRI for cartilage damage.

**Figure 8:** Contrast-to-noise ratio CNR of cartilage to surrounding tissue in different sequences.

**Figure 9:** Comparison of sensitivity and specificity.

**Figure 10:** Comparison of cartilage *T*2 values.

**Table 1:** Differences in BIM.

Partition	Low (<18.5)	Medium (18.5–24)	High (>24)
Patellar cartilage	123.11 ± 243.42	52.32 ± 255.10	−43.15 ± 344.32
Medial femoral condyle cartilage	35.42 ± 24.13	−32.13 ± 350.33	35.13 ± 224.43
Lateral femoral condyle cartilage	24.43 ± 35.34	−30.23 ± 313.21	12.35 ± 233.52
Lateral tibial plateau cartilage	−10.41 ± 25.31	−33.22 ± 15.52	−10.55 ± 134.44

**Table 2:** ICC test results.

Partition	ICC	*P*
Patellar cartilage	0.950	0.000
Medial femoral condyle cartilage	0.849	0.007
Lateral femoral condyle cartilage	0.759	0.044
Lateral tibial plateau cartilage	0.775	0.045

**Table 3:** Characteristics of magnetic resonance imaging in different knee injury sites.

Injured area	Sensitivity (%)	Specificity (%)
ACL	88.4	89
PCL	100	100
Meniscus	82	84
Collateral ligament	84	89

**Table 4:** Different degrees of injury in the left and right patellar cartilage regions of athletes.

Average *T*2 value (*T*2av) (ms)	Right patellar cartilage	Left patellar cartilage
Medial region	40.01 ± 3.88	39.65 ± 3.46
Central district	40.24 ± 4.79	39.99 ± 4.19
Lateral area	42.66 ± 5.09	41.33 ± 4.39
Outer zone	43.55 ± 5.38	41.22 ± 4.11

**Table 5:** Comparison of the average *T*2 value (*T*2av) of the left and right patellar cartilage between the sports trauma group and the control group.

Average *T*2 value (*T*2av) (ms)	Right patellar cartilage	Left patellar cartilage
Sports trauma group	42.28 ± 5.26	38.82 ± 4.68
Control group	35.63 ± 4.26	35.32 ± 3.86
*t*	6.26	6.82

**Table 6:** Preoperative lysholm score.

Group	Injured days	Number of sprains (times)	Preoperative lysholm score
*A*	0	0.00	47
*B*	18	1.8 ± 1.1	52
*P*	0.018	0.00	0.005

## Data Availability

The datasets generated during and/or analyzed during the current study are not publicly available due to sensitivity and data use agreement.
